# The Research on the Impact of Management Level’s Charismatic Leadership Style on Miners' Unsafe Behavior

**DOI:** 10.2174/1874120701509010244

**Published:** 2015-09-17

**Authors:** Hongxia Li, Hongxi Di, Shuicheng Tian, Jian Li

**Affiliations:** 1 School of Management, Xi’an University of Science and Technology, Xi’an, 710054, China; 2 School of Energy Engineering, Xi’an University of Science and Technology, Xi’an, 710054, China; 3 Key Laboratory of Western Mine Exploitation and Hazard Prevention, Ministry of Education, Xi’an University of Science and Technology, Xi’an, 710054, China; 4 Shanxi Provincial AuditOffice, Xi’an, 710054, China

**Keywords:** Charismatic leadership style, coal mine workers, structural equation model, unsafe behavior

## Abstract

The aim of this study is research the impact of management level’s charismatic leadership style on miners' unsafe behavior by using the questionnaires on charismatic leadership style, safety attitude and the miners' unsafe behavior measurement to investigate 200 employees in Shen Dong Company. The research results suggest that management level’s charismatic leadership style have very important influence on miners' unsafe behavior and the influence is affected by the safety attitude which is the intermediary function. In the end, this study propose advice on how to improve the coal mine enterprise managers charismatic leadership style in the coal mine enterprise's safety management work, including attach great importance to a variety of incentive methods, set up safety moral models, practice of inductive leadership concept, create a good atmosphere of safety, etc for reference for coal mining enterprises.

## 1. INTRODUCTION

In recent years, the “Charismatic Leadership” Theory has aroused increasingly great attention in business and academic circles. The charismatic leadership model by House [1] was built based on following models. Charismatic leaderships usually have the power of role models and serve as good examples advocating some beliefs and values if they hope that their followers hold these beliefs and values; charismatic leaderships are competent in some fields; they set clear goals with moral colors; they have high expectations for their followers and believe that their followers have the ability to do what they are expected to do. As a result, such behaviors increase the understanding of followers towards their own abilities and efficacy, thus further improving their performance. According to Bass and Avolio [2], charismatic leaderships have following features. Charismatic leaderships can usually stir enthusiasms of followers for work and make them have particularly high expectations, so that charismatic leaderships can motivate followers while achieving organizational goals; charismatic leaderships adhere to an independent way of thinking and create a good atmosphere to support their followers; charismatic leaderships usually pay great attention to intellectual excitation of their followers including the belief and core value development in organizational development; charismatic leaderships fully show their charm, to motivate their followers to pursue goals they develop, set a good example and win recognition of followers, so that followers have a sense of mission for their self-development. Thus it can be seen that leaderships serve as instructors and give relevant advices.

## 2. THEORIES AND RESEARCH HYPOTHESES

In a paper, Bao Lingling and Wang Tao [3] investigate the impact of charismatic leaderships on subordinates in China from three dimensions. The first one is the personality charm; the second one the ability charm; the third one relationship charm. Based on an empirical study, Feng Jiangping and Luo Guozhong [4] reveal that charismatic leadership is a five-factor models. Based on a questionnaire survey, an exploratory factor analysis is made and five factors are chosen from seven kinds of traits for validations. 

In research on unsafe behaviors made abroad, both Senders [5] and Themse [6] give definitions to human error. In China, Zhou Gang [7] also makes research on human error and unsafe behaviors. In general, human error refers to the phenomenon that behavioral results of humans deviate from specified targets or exceed acceptable limits, thus producing a negative impact. In analyzing fatal accidents, unsafe behaviors are defined as human behavioral errors which may cause accidents. Unsafe behaviors refer to behavioral errors of individuals that can cause accidents. To be specific, unsafe behaviors refer to people’s non-compliance with provisions of the production, operating provisions and operating methods in production which would incur a series of security risks. 

According to Cao Qingren, unsafe behaviors refer to human behaviors that once caused or may cause accidents and the direct cause of accidents [8]. According to research made at home and abroad on operation modes of people, it can be seen that the majority of scholars believe that human causes can be equated to unsafe behaviors of human. Li Kai [9] divides unsafe operating behaviors into unintentional and intentional ones, from the perspective of cognitive psychology. 

In the field of security management, Barling [10] and other scholars believe that transformational leadership can effectively improve the safety level of employees. Du Fengwen [11] concludes that charismatic leadership has a significant impact on organizational citizenship behaviors, on the basis of the Achievement Motivation Theory, the Organizational Citizenship Behaviors, and the Charismatic Leadership Theory. 

However, few studies have been made on the impact of charismatic leadership management in coal mine enterprises on unsafe behaviors of miners. Miners, constituting the core part of the development of coal mine enterprises, have received increasingly great attention from coal mine enterprises. Meanwhile, safety problems, enjoying the top priority in safety production of miners, have attracted more and more attention from coal mine enterprises. Effective measures should be adopted to prevent and control unsafe behaviors of miners, as their behaviors are of great significance for the safety production of enterprises. 

According to research on relationships between leadership styles and behaviors of employees, attitudes towards safety, as a mediator between leadership behaviors and employee behaviors, has a certain inherent impact on mentality of miners, thus further affecting behaviors of miners at work. Donald & Young [12] think that there is a significant correlation between attitudes towards safety and safe behaviors, and changes in attitudes towards safety can effectively improve the safety performance of an organization. According to Li Naiwen [13], each dimension of transformational leadership has a significant impact on safety performance of employees and employees’ attitudes towards safety serve as a mediator between each dimension of transformational leadership and safety performance of employees. Conclusions made by Li Naiwen theoretically support the idea that grass-roots transformational leadership can effectively improve safety performance of employees. 

In this paper, based on domestic and overseas research and theoretical analyses made of impacts of charismatic leadership on unsafe behaviors of miners, a theoretical analysis is made of impacts of four dimensions of charismatic leadership including Charisma, Incentive & Care, Visionary Appeal and Moral Example on unsafe behaviors of miners, and research hypotheses are presented. Moreover, the role of attitudes towards safety as a mediator between charismatic leadership and unsafe behaviors of miners is analyzed. On this basis, the research model for this paper, that is, the model for impacts of charismatic leadership on unsafe behaviors of miners is developed to investigate impacts of charismatic leadership on unsafe behaviors of miners. In this research model, charismatic leadership is an explanatory variable while unsafe behaviors of miners serve as an explained variable. Attitudes of miners towards safety produce mediating effects on impacts of charismatic leadership on unsafe behaviors of miners. 

The model built for this research is shown in Fig. (**1**).

## 3. RESEARCH METHODS

### 3.1 Measurement

Measurement of background variables: background variables include the gender, age, type of work, education background and working company and so on. 

Measurement of Leadership styles: Cheung and other scholars study the SLB scale on the basis of the MLQ research made by Bass. Zhou, Wang and Jiang use this scale to verify the relationship between charismatic leadership and ERP performance and make an in-depth study to find that Cronbach’α in this scale is greater than 0.70. In this paper, the scale which is modified by Zhang Zhijie [14] on the basis of charismatic leadership developed by Cheung is used as a reference. This scale, whose Cronbach’α is greater than 0.70, shows high reliability and validity and has four dimensions including charismas, incentives & care, visionary appeal and moral example. The four dimensions include 6, 6, 4 and 4 items, respectively. The Likert Scale is used for scoring points. The Cronbach’α is 0.853.

Measurement of attitudes towards safety: attitudes towards safety are measured through a scale which is adapted based on the self-made scale by Wu Jieliang [15] and Li Naiwen and Huang Peng [16]. Measurement indexes for attitudes towards safety mainly include awareness of the importance of safety operation and individual tendencies to see safety. Based on the two measurement indexes and relevant literature, the first draft of questionnaire for investigating attitudes towards safety is developed, including 3 items. The Likert Scale is used for scoring points. The Cronbach’α is 0.869.

Measurement of unsafe behaviors: in this paper, on the basis of research achievements made by Wu Jianjin [17], Zheng Ying [18] and other scholars and field research made on coal mine enterprises, typical unsafe behaviors of miners are taken as indictors to measure unsafe behaviors of miners. Three indicators are used for measuring unsafe behaviors, including safety inspection before work, rules and regulations breaking at work and safety production at work and covering three items. The Likert Scale is used for scoring points and the Cronbach’α is 0.7.

### 3.2 Research Samples

Respondents are from 4 coal mines of the SD Company. A total of 200 copies of questionnaires were sent out and 190 copies were received. The response rate of questionnaires was 91.30%. 179 valid questionnaires were obtained, after questionnaires of respondents who omitted some questions or gave the same option for all questions were eliminated. The validness rate of questionnaires received was 89.5%. Among 179 respondents completing valid respondents, 126 of them are aged 35 or under; 20 of them are aged 36 to 40; 21 of them are aged 41 to 45; 22 of them are aged over 45. In terms of education backgrounds, 44 of them were graduated from middle schools or primary schools or even received no education; 88 of them were graduated from high schools; 23 of them were graduated from institutions of higher education, 18 of them have bachelor degrees; 10 of them have master or PHD degrees. In terms of in-service years, 76 of them have worked for no more than 5 years; 52 of them have worked for 6 to 10 years; 23 of them have worked for 11 to 20 years; 28 of them have worked for over 20 years. In terms of posts of duty, 46 of them are responsible for dig-in; 35 of them are responsible for coal mining; 42 of them are coal heavers; 39 of them are responsible for electromechanical guarantees; 17 of them are responsible for ventilations. 

### 3.3 Moeel Fitting Test

In order to further explore impact of each dimension of charismatic leadership on unsafe behaviors of miners, firstly, a theoretical model for impacts of charismatic leadership on unsafe behaviors of miners is built. Secondly, Amos7.0 and the maximum likelihood method are used to examine hypotheses based on this theoretical model, thus obtaining the goodness of fit for this model. Lastly, the model is modified on the basis of model operation results. The hypothesis that i has no significant impact is eliminated and the final model is built, as shown in Fig. (**2**).

Fitting results of the final model are shown in Table **1**. Values of χ^2^/df and RMSEA are respectively 2.776 and 0.041 which are less than 3 and 0.10 as required values. Both NFI and IFI are greater than 0.90 as the required value. Although CFI fails to reach 0.9, it is quite approximate to 0.9. It indicates that the absolute model fitting effects are raised to the normalized and required level. Regression coefficients and statistical testing results of the model are shown in the following Table **1**.

### 3.4 Anlysis of Relationgships between Various Variables in Model

In Table **2**, path relationships between structural latent variables of the final model and their error parameter values are shown. According to data, the absolute value of the variable parameter C.R is greater than 2.391 and less than 5.359. Both 2.391 and 5.359 are much greater than 1.96 as the normalized value. As normative standards for each error term are small in number, significance is tested to be up to standards.

7Standardized path coefficients between charismatic leadership in coal mine management and unsafe behaviors of miners are listed in Table **2**. As it is proved by the structural equation model, among 9 hypotheses presented above, 7 of them are supported while 2 of them are not supported. Influence paths between incentives & care and visionary appeal as two dimensions of charismatic leadership and unsafe behaviors fail to be supported. However, incentives & care and visionary appeal exert indirect impacts on unsafe behaviors of employees through attitudes towards safety. 

Occurrence of unsafe behaviors in coal mines as an endogenous latent variable are affected charisma, incentives & care, visionary appeal and moral examples of leaderships as four exogenous latent variables. 

According to test analytical results of the structural equation, it can be seen that standardized path coefficients between moral example and charisma as exogenous latent variables and unsafe behaviors as an endogenous variable are respectively -0.32 and -0.28, indicating that moral example and charisma are negatively correlated to unsafe behaviors. 

Moral example, incentives & care, visionary appeal and charisma as exogenous latent variables have a negative impact on unsafe behaviors through attitudes towards safety as a mediator. The standardized path coefficient between attitudes towards safety and unsafe behaviors is -0.43;

Standardized path coefficients between Incentives & care and visionary appeal and attitudes towards safety as a mediator are respectively 0.39 and 0. 41. It indicates that although Incentives & care and visionary appeal are not directly related to the occurrence of unsafe behaviors, they have significantly positive correlations with attitudes towards safety. Employees’ attitudes towards safety can be effectively improved by increasing incentives & care and visionary appeal, in order to reduce unsafe behaviors. Therefore, it can be concluded that each dimension of charismatic leadership has a negative impact on unsafe behaviors of miners. 

As can be seen from the above analysis, attitudes towards safety serve as a mediator between charismatic leadership and unsafe behaviors of miners. The standardized path coefficient between moral example and attitudes towards safety is 0.49 while that between moral example and unsafe behaviors is -0.32. It indicates that the better the exemplary role of the corporate management is, the better employees’ attitudes towards safety would be. In this way, unsafe behaviors of employees can be effectively reduced. 

The same is true with charisma as another dimension of charismatic leadership. Charisma also has a negative impact on unsafe behaviors. The standardized path coefficient between unsafe behaviors and charisma is -0.28, indicating that charisma of the corporate managements has a negative impact on unsafe behaviors, and the greater the impact of charisma on employees is, the lower the possibility that employees make unsafe behaviors would be.

## 4. CONCLUSIONS AND RECOMMENDATIONS

In the field of safety management, many scholars at home and abroad have made research on the role of charismatic leadership in security management of enterprises. However, no scholar has taken attitudes towards safety as a mediator to investigate deep-seated impacts of charismatic leadership on unsafe behaviors of miners. In this paper, the structural equation and relevant theories are used to make a scientific discussion of impacts of charismatic leadership on unsafe behaviors of miners, based on survey data about large-sized coal mine enterprises. Following conclusions are drawn. 

(1) Charismatic leadership has a significantly negative impact on unsafe behaviors of miners. Moral example, charisma, incentives & care and visionary appeal as four dimensions of charismatic leadership have a negative impact on unsafe behaviors of miners. They affect unsafe behaviors of miners, in varying degrees. If the four dimensions are sorted according to their influence degrees on unsafe behaviors from the higher to lower, the order is: moral example, charisma, incentives & care and visionary appeal. 

(2) Attitudes towards safety produce indirect effects on relationships between charismatic leadership and unsafe behaviors of miners, thus indirectly affecting the impact of charismatic leadership on unsafe behaviors of miners. If the four dimensions are sorted according to the size of indirect effects of attitudes towards safety on relationships between each dimension and unsafe behaviors of miners from the larger to smaller, the order is: moral example, incentives & care, charisma and visionary appeal. 

(3) Coal mine enterprises should pay great attention to the role of charismatic leadership in coal mine safety management and further improve the leadership charisma by means of adopting effective incentive, applying some leadership theories, building security visions, strengthening human care and attaching great importance to leadership as moral models, in hope of effectively preventing and controlling unsafe behaviors of miners.

## Figures and Tables

**Fig. (1):** Research model for impacts of charismatic leadership on unsafe behaviors of miners. Based on the theoretical analysis made above, following hypotheses are presented and examined. H 1: Incentive & care has a negative impact on unsafe behaviors of miners. H 2: Visionary appeal has a negative impact on unsafe behaviors of miners. H 3: Charisma has a negative impact on unsafe behaviors of miners. H 4: Moral example has a negative impact on unsafe behaviors of miners. H 5: Incentive & care has a positive impact on miners’ attitudes towards safety. H 6: Visionary appeal has a positive impact on miners’ attitudes towards safety. H 7: Visionary appeal has a positive impact on miners’ attitudes towards safety. H 8: Moral example has a positive impact on miners’ attitudes towards safety. H 9: Attitudes towards safety has a positive impact on miners’ unsafe behaviors.

**Fig. (2):** Final fitting model for relationships between charismatic leadership unsafe behaviors.

**Table 1.** Statistical values of goodness of model fit after indexes are eventually modified.

χ^2^/df	RMSEA	NFI	IFI	CFI
2.776	.041	.901	.912	.887

**Table 2.** Path parameter estimation for the final model.

Path relationships between various variables			Standardized estimation	Non-standardized estimation	Standard error	Critical value	P value
Attitudes towards safety	<---	Moral example	.490	.480	.088	5.475	***
Attitudes towards safety	<---	Incentives & care	.387	.334	.102	3.794	***
Attitudes towards safety	<---	Charisma	.413	.323	.112	3.688	***
Attitudes towards safety	<---	Visionary appeal	.253	.193	.053	-4.774	.004
Unsafe behaviors	<---	Attitudes towards safety	-.432	-.376	.107	-4.420	***
Unsafe behaviors	<---	Moral example	-.315	-.294	.059	-5.339	.003
Unsafe behaviors	<---	Charisma	-.283	-.204	.047	-6.021	***
